The article "Association of TCM body constitution with insulin resistance and risk of diabetes in impaired glucose regulation patients" was published in 2017. Journal: BMC Complement Altern Med.

# Association of TCM body constitution with insulin resistance and risk of diabetes in impaired glucose regulation patients

**DOI:** 10.1186/s12906-017-1964-0

**Published:** 2017-09-11

**Authors:** Hong You, Tong Zhang, Wen Feng, Yun Gai

**Affiliations:** Seventh People’s Hospital of Shanghai University of TCM, No.358 Datong Road, Gaoqiao Town, Pudong New District, Shanghai, 200137 China

**Keywords:** Impaired glucose regulation (IGR), Traditional Chinese medicine (TCM), Body constitution, Diabetes mellitus (DM), Insulin resistance, Inflammatory response

## Abstract

**Background:**

Impaired glucose regulation (IGR) patients have increased risk of type 2 diabetes mellitus (T2DM). Identifying relevant risk factors in IGR subjects could facilitate early detection and prevention of IGR progression to diabetes. This study investigated the association between Traditional Chinese Medicine (TCM) body constitution and serum cytokines, and whether body constitution could independently predict diabetes in IGR subjects.

**Method:**

Patients with IGR (*n* = 306) received a blood test and their body constitution type was assessed using a body constitution questionnaire (BCQ). Serum levels of cytokines were measured by ELISA. Patients were followed up for at least three years, and their status of diabetes were recorded. Multivariate logistic regression was used to estimate odds ratios (ORs) of diabetes for body constitution.

**Results:**

Phlegm-damp, Damp-heat and Qi-deficiency were three most common unbanlenced constitutions among IGR subjects. Phlegm-damp and Damp-heat constitution subjects showed higher serum levels of interleukin 6 (IL-6), tumour necrosis factor-α (TNF-α), leptin and lower serum levels of adiponectin (P<0.05). Qi-deficiency constitution subjects showed higher serum levels of leptin and lower serum levels of adiponectin, glucagon-like peptide-1 (GLP-1) and gastric inhibitory polypeptide (GIP) (P<0.05). Subjects with Phlegm-damp or Damp-heat constitution demonstrated a significantly higher risk of diabetes (P<0.05).

**Conclusion:**

Phlegm-damp and Damp-heat TCM body constitution are strongly associated with abnormal serum cytokines, and could potentially serve as a predictor of diabetes in IGR subjects. Body constitution can help to identify IGR subjects who are at a high risk of progression to diabetes.

## Background

Diabetes mellitus (DM) is a chronic metabolic disease with rapidly increasing incidence, and its global prevalence is estimated to reach over 552 million by 2030 [1]. Impaired glucose regulation (IGR) is an intermediate metabolic state between normal glucose regulation and diabetes mellitus, including impaired fasting glucose (IFG) and impaired glucose tolerance (IGT), also known as pre-diabetes mellitus (pre-DM) [2]. About 9 % of IGR patients could progress to diabetes mellitus in a mean time of 34 months [3]. IGR is considered to be a high-risk factor for cardiovascular disease (CVD), stroke and associated death [4, 5]. Insulin resistance is one important mechanism underlying diabetes mellitus and progression to diabetic vascular complications and cardiovascular disease [6]. Moreover, insulin resistance exists in IGR subjects and is associated with unfavorable cardiac structure and function before the development of diabetes mellitus [7, 8]. Therefore, inhibition of insulin resistance is a key treatment strategy for IGR patients to prevent the progression of diabetes mellitus. The pathogenesis of IGR and diabetes is multifactorial, thus it is urgent for early detection of IGR cases with higher risk to progression to diabetes.

Traditional Chinese Medicine (TCM) is a kind of complementary and alternative medicine (CAM) and performs personalized therapy based on body constitution (BC) theory [9, 10]. TCM body constitution refers to an integrated, metastable and natural specialty of individuals in morphological structures, physiological functions, and psychological status, formed on the basis of congenital and acquired endowments in the process of life [11]. TCM constitutions determine the individual’s specificity [12], and thus influence not only the susceptibility to diseases but also the progression and prognosis of diseases [13]. TCM practitioners performe personalized treatment and prevention according to body constitution of each individual, thereby achieving optimal health promotion effects [14, 15].

TCM body constitution is divided into balanced constitution also nine types known as Neutral constitution, Qi-deficiency constitution, Yang-deficiency constitution, Yin-deficiency constitution, Phlegm-damp constitution, Damp-heat constitution, Blood-stagnation constitution, Qi-stagnation constitution and Special diathesis constitution. Neutral constitution is a balanced constitution and represents an overall healthy state, while people with other eight unbalanced constitutions are prone to certain diseases.

Therefore, the present study aimed to investigate the association between TCM constitutional types and insulin resistance and incidence of deabetes in IGR patients. Our results could help identifying IGR subjects with high risk for daibetes and help clinicians focus preventive strategy more effectively on these patients.

## Methods

### Study design and subjects

We conducted this prospective study form January 2011 to June 2012 at the Department of Diabetes of Seventh People’s Hospital of Shanghai University of TCM. A total of 306 individuals diagnosed with IGR were included, with a median age of 56 years old and 155 males and 155 females. Every subject received oral glucose tolerance test (OGTT) and the fasting blood glucose and 2-h blood glucose were measured. The IGR was defined as fasting blood glucose between 6.1 and 6.9 mmol /L, and 2-h blood glucose < 7.8 mmol /L; or fasting blood glucose < 6.1 mmol /L, and 2-h blood glucose between 7.8 and 11.0 mmol /L. The age, sex, body mass index (BMI), and lifestyle were collected, and TCM body constitution was measured. The inclusion criteria were the following: ① Shanghai locals; ② 40 to 70 years of age; ③ Voluntary cooperation with investigation. The exclusion criteria were the following: ① IGR secondary to other diseases; ② Subjects who complicated with cardiovascular or cerebralvascular diseases; ③ Subjects with diseases of kidney, blood or immune system; ④ Patients with severe water and electrolyte disturbances or mental disorders. All subjects were followed up for at least three years, and their fasting and 2-h blood glucose was measured to monitor the occurrence of diabetes. The diabetes was defined as fasting blood glucose ≥7.0 mmol /L, or 2-h blood glucose ≥11.1 mmol /L. This study protocol was approved by the Institutional Review Board of Seventh People’s Hospital of Shanghai University of TCM. A signed written informed consent was obtained by all patients to participate in this study and publish this manuscript. A total of 448 participants with IGR were recruited in the study, and 306 participants were included in the final analysis (Fig. 1).

**Fig. 1:** The recruitment flowchart of the study participants. A total of 448 participants with IGR were recruited in the study, 395 cases were evaluated by BCQ for their TCM body constitutions, 352 cases were performed follow-up, and 306 cases were included in the final analysis

### Measurement of TCM constitution types

The body constitution status of all the participants was evaluated using the TCM Physical Constitution Scale [16]. The scale consists of 60 items scored on a 5-point scale, ranging from 1 (not at all) to 5 (very much) (Appendix). It has nine subscales which assess one type of TCM constitution individually, including Neutral constitution, Qi-deficiency constitution, Yang-deficiency constitution, Yin-deficiency constitution, Phlegm-damp constitution, Damp-heat constitution, Blood-stagnation constitution, Qi-stagnation constitution and Special diathesis constitution. For each item, subjects selected one from five answers (Not at all, few, sometimes, often, always), and gvien a respevtive score (1–5). For each subscale, the original score was first calculated by summing of the scores for each item). The derived score of each subscale was calculated from the following formular: (original score-the possible lowest score of the subscale)/(possible highest score-possibl lowest score) × 100, ranging from 0 to 100 points. Neutral constitution referred to the patients with derived scores of the eight unbalanced constitutions being <40 points, and the derived score of the Neutral constitution being ≥60 points. If the score of any constitution subscale was ≥40 points, unbalanced constitutions were diagnosed. Patients with two or more constitutional types ≥40 points, subjects were diagnosed with constitution of the highest subscale score.

### Determination of clinical data and laboratory parameters

The following variables were recorded for each IGR patient: age, gender, body mass index (BMI), fasting plasma insulin (FPI), total cholesterol (TC), triglyceride (TG), serum creatinine (Scr) and blood urea nitrogen (BUN). The presence of diabetes at three years was used as the endpoint. Blood samples were collected from IGR patients with at admission to our hospital.

### Determination of serum cytokines levels

Enzyme-linked immunosorbent assay (ELISA) was performed to determin the serum levels of interleukin 6 (IL-6), tumour necrosis factor-α (TNF-α), adiponectin, leptin, glucagon-like peptide-1 (GLP-1) and gastric inhibitory polypeptide (GIP). Venous blood samples were collected from each subjects at admission to our hospital, and after centrifugation at 1000 g for 15 min, the serum was separated and stored in aliquots at −70 °C. The serum IL-6, TNF-α, adiponectin, leptin, GLP-1 and GIP were measured by ELISA kit (R&D Systems, Minneapolis, MN; cat. no. DY720), according to the manufacturer’s protocol. The absorbance at OD450 wavelength was measured by an ELISA plate reader (Ricso RK201, Shenzhen Ricso Technology Co., Ltd., Shenzhen, Guangdong, China). The serum concentrations insulin resistance factors were determined by the standard curves constructed from counterpart recombinant human protiens.

### Statistical analysis

The statistical analysis was performed with SPSS 19.0 (SPSS Inc., Chicago, IL, USA). The data were presented as medians and interquartile ranges for continuous variables and as frequencies and percentages for categorical variables. Differences between groups of categorical variables were compared using a chi-square test, and differences between groups continuous variables were compared using Wilcoxon-Mann-Whitney test. Multiple logistic regression analysis was performed to calculate the odds ratios (ORs) and determine the independent contribution of risk fartors. A probability value of P<0.05 was considered as statistically significant difference.

## Results

### Characteristics of the patients

A total of 306 participants who completed the questionnaires and 3-year follow-up were included in the analyses. The study group included 165 (53.9%) males and 141 (46.1%) females with a median age of 52 years. After three-year follow-up, there were 56 (18.3%) subjects diagnosed with diabetes.

### TCM constitutional types

Among these 306 cases, there were 57 cases of Phlegm-damp constitution (18.6%), 52 of Damp-heat constitution (17.0%), 47 of Neutral constitution (15.4%), 39 of Qi-deficiency constitution (12.7%), 33 of Yin-deficiency constitution (10.8%), 28 of Blood-stagnation constitution (9.2%), 24 of Yang-deficiency constitution (7.8%), 21 of Qi-stagnation constitution (6.9%) and 5 of Special diathesis constitution (1.6%). Subjects with Qi-deficiency constitution had significantly higher BMI, FPI, TC and TG (P<0.05). Subjects with Phlegm-damp or Damp-heat constitution had significantly higher BMI, TC, TG, Scr and BUN (P<0.05) (Table 1).

**Table 1:** Patients’ characteristics

	Age	Male (%)	BMI (Kg/m^2^)	FPI (mu/L)	TC (mmol/L)	TG (mmol/L)	Scr (μmol/L)	BUN (mg/dL)
Qi-deficiency								
Yes (*n* = 39)	52 (49–54)	18 (46.2)	27.7 (26.3–28.9)	14.3 (13.1–16.3)	5.3 (4.8–5.8)	2.5 (2.3–2.7)	113 (96–133)	14.0 (12.6–15.7)
No (*n* = 267)	52 (49–55)	147 (55.1)	26.9 (25.4–28.1)	13.5 (11.8–15.9)	4.8 (4.1–5.5)	2.3 (1.8–2.8)	110 (93–126)	113.8 (12.9–15.1)
*P* value	0.825	0.308	0.026	0.030	0.002	0.011	0.482	0.627
Phlegm-damp								
Yes (*n* = 57)	52 (49–55)	34 (59.6)	27.3 (26.0–28.8)	14.7 (12.6–16.5)	5.2 (4.6–5.6)	2.5 (2.2–2.8)	117 (100–137)	14.6 (13.4–15.5)
No (*n* = 249)	52 (49–55)	131 (52.6)	26.9 (25.4–28.1)	13.6 (11.8–15.8)	4.8 (4.1–5.5)	2.3 (1.8–2.7)	109 (92–125)	13.8 (12.8–14.9)
P value	0.640	0.378	0.029	0.054	0.014	0.029	0.024	0.013
Damp-heat								
Yes (*n* = 52)	51 (48–54)	31 (59.6)	27.6 (26.5–28.6)	14.9 (13.1–16.4)	5.3 (4.6–5.7)	2.5 (2.2–2.9)	118 (109–135)	14.7 (13.2–15.5)
No (*n* = 254)	52 (49–55)	134 (52.8)	26.8 (25.3–28.2)	13.5 (11.8–15.8)	4.8 (4.1–5.5)	2.3 (1.8–2.7)	108 (89–125)	13.8 (12.8–14.9)
P value	0.081	0.446	0.013	0.021	0.029	0.010	0.001	0.018

Categorical Variable are expressed as frequency (%) and analyzed by Chi-squared test (Sex); Continuous variable are expressed as median (25th to 75th percentiles) and analyzed by Mann-Whitney U test

*BMI* body mass index, *FPI* fasting plasma insulin, *TC* total cholesterol, *TG* triglyceride, *Scr* serum creatinine, *BUN* blood urea nitrogen

### Associations of body constitution with insulin resistance factors

To evaluate the associations of TCM constitutional types with insulin resistance, we compared serum levels of IL-6, TNF-α, adiponectin, leptin, GLP-1 and GIP in patient subgroups dividing by the presence of TCM constitutional types, including Qi-deficiency constitution, Phlegm-damp constitution and Damp-heat constitution. Serum levels of IL-6 and TNF-α were significantly higher in subjects with Phlegm-damp constitution and subjects with Damp-heat constitution (Fig. 2). Decreased serum levels of adiponectin and increased serum levels of leptin were shown in subjects with Qi-deficiency constitution, subjects with Phlegm-damp constitution and subjects with Damp-heat constitution (Fig. 3). Serum levels of GLP-1 and GIP were significantly lower in subjects with Qi-deficiency constitution (Fig. 4).

**Fig. 2:** Serum levels of inflammatory mediators in IGR subjects with TCM body constitutions. Serum levels of IL-6 and TNF-α were measured by ELISA, and their associations with Phlegm-damp (**a, d**), Damp-heat (**b, e**) and Qi-deficiency (**c, f**) were investigated. Serum IL-6 and TNF-α levels are significantly higher in IGR subjects with Phlegm-damp or with Damp-heat constitutions as compared with IGR subjects without respective constitutions. Box plots are displayed, where the bold black line indicates the median per group, the box represents 50% of the values, and horizontal lines show minimum and maximum values of the calculated non-outlier values; open circles indicate outlier values. Wilcoxon-Mann-Whitney test was performed. *P<0.05. IGR: impaired glucose regulation; IL-6: interleukin 6; TNF-α: tumour necrosis factor-α

**Fig. 3:** Serum levels of adiponectin and leptin in IGR subjects with TCM body constitutions. The associations of adiponectin and leptin with Phlegm-damp (**a, d**), Damp-heat (**b, e**) and Qi-deficiency (**c, f**) were investigated. Serum adiponectin levels are significantly lower in IGR subjects with Phlegm-damp, Damp-heat and Qi-deficiency constitutions as compared with IGR subjects without respective constitutions, while serum leptin levels are significantly higher all three TCM constitution types.Wilcoxon-Mann-Whitney test was performed. *P<0.05. IGR: impaired glucose regulation

**Fig. 4:** Serum levels of gut hormones in IGR subjects with TCM body constitutions. The associations of GLP-1 and GIP with Phlegm-damp (**a, d**), Damp-heat (**b, e**) and Qi-deficiency (**c, f**) were investigated. Serum GLP-1 and GIP levels are significantly lower in IGR subjects with Qi-deficiency as compared with IGR subjects without Qi-deficiency. Wilcoxon-Mann-Whitney test was performed. *P<0.05. IGR: impaired glucose regulation; GLP-1: glucagon-like peptide-1; GIP: gastric inhibitory polypeptide

### Incidence of diabetes in IGR patients according to body constitution

Among all the 306 study participants, 56 (18.3%) cases developed diabetes in three years. There were 18 cases of diabetes among 57 subjects with Phlegm-damp constitution, 17 diabetes among 52 subjects with Damp-heat constitution, 3 diabetes among 47 subjects with Neutral constitution, 8 diabetes among 39 of Qi-deficiency constitution, 1 diabetes among 33 subjects with Yin-deficiency constitution, 2 diabetes among 28 subjects with Blood-stagnation constitution, 4 diabetes among 24 subjects with Yang-deficiency constitution, 2 diabetes among 21 subjects with Qi-stagnation constitution and 1 diabetes among 5 subjects with Special diathesis constitution. There were significant difference between diabetes incidence among different body constitutions (*P* = 0.001), with Phlegm-damp, Damp-heat and Qi-deficiency constitutions showing the highest probability of developing diabetes. Then the incidence of diabetes was compared between different body constitution types. Participants with Phlegm-damp or Damp-heat had significantly higher incidence of diabetes (31.6% versus 15.3%, *P* = 0.007; 32.7% versus 15.4%, *P* = 0.005) (Table 2). There was no significant differenc in incidence of diabetes between Participants with Qi-deficiency and without Qi-deficiency.

**Table 2:** Incidence of diabetes in IGR patients according to BC

	Diabetes	Nondiabetes	P value
Qi-deficiency			
Yes (n = 39)	8 (20.5%)	31 (79.5%)	0.662
No (n = 267)	48 (18.0%)	219 (82.0%)	
Phlegm-damp			
Yes (n = 57)	18 (31.6%)	39 (68.4%)	0.007
No (n = 249)	38 (15.3%)	211 (84.75)	
Damp-heat			
Yes (n = 52)	17 (32.7%)	35 (67.3%)	0.005
No (n = 254)	39 (15.4%)	215 (84.6%)	

Categorical Variable are expressed as frequency (%) and analyzed by Chi-squared test

### TCM body constitution may be a predictive factor for diabetes

To evaluate whether TCM body constitution is an independent predictive factor of diabetes, we performed multivariate logistic regression analysis. Participants with Phlegm-damp or Damp-heat were more likely to develop diabetes in three years (Phlegm-damp: OR = 2.846, 95% CI = 1.345–6.022, *P* = 0.006; Damp-heat: OR = 3.080, 95% CI = 1.443–6.574, *P* = 0.004). In addition, FPI, TC and Scr were also significantly associated with diabetes in three years (Table 3).

**Table 3:** Multiple logistic regression analysis of variables to predict diabetes

Variable	Odds Ratio	95% Confidence Interval	P value
FPI	1.133	1.016 to 1.264	0.025
TC	1.430	1.017 to 2.011	0.039
Scr	1.014	1.001 to 1.026	0.032
Phlegm-damp	2.846	1.345 to 6.022	0.006
Damp-heat	3.080	1.443 to 6.574	0.004

Multiple logistic regression analysis was performed to calculate the odds ratios

*FPI* fasting plasma insulin, *TC* total cholesterol, *Scr* serum creatinine

## Discussion

TCM body constitution could indicate the overall health status of individuals, and unbalanced body constitution often represents deteriorated health status, a condition that western medicine will diagnose as “no disease”. Therefore, body constitution has enormous potential application in preventive treatment of diseases. Impaired glucose regulation (IGR) is an intermediate metabolic state between health status and diabetes mellitus, and is a potential illness for the research and clinical application of body constitution. This study explored TCM body constitution types among IGR subjects and their associations with serum cytokines and incidence of diabetes. This is the first investigation on the association between TCM body constitution type and risk factors of daibetes among IGR subjects. The results showed that Phlegm-damp, Damp-heat and Qi-deficiency constitution were all associated with lower serum level of adiponectin and higher serum level of leptin. Phlegm-damp and Damp-heat constitution subjects showed higher serum levels of IL-6 and TNF-α, while Qi-deficiency constitution subjects showed lower serum levels of GLP-1 and GIP. Subjects with Phlegm-damp or Damp-heat constitution demonstrated a significantly higher risk of diabetes. The findings of this study would help TCM professionals to identify IGR subjects who are at a high risk of progression to diabetes, thus proving focused therapy base on these unbanlenced body constitution.

The findings of the present study showed that more than 80 % of IGR subjects had unbalanced TCM constitution, and this indicates that they were in the deteriorated health state. The most common unbalanced TCM constitution types among the IGR subjects were Phlegm-damp, Damp-heat and Qi-deficiency. Our results are in consistent with that of a previous investigation conducted in Shanghai, Nanjing, Hangzhou and Qingdao, which involved 1590 metabolic syndrome (MS) patients and found that Phlegm-damp, Damp-heat and Qi-deficiency were the three dominant constitutional types in the MS patients [17]. However, the finding of our study differed from previous investigation which reported that dominant unbalanced TCM constitution types were Yang deficiency, Yin deficiency and Phlegm stasis [18]. The difference may probably be caused by differences in samples, and our study involved IGR while their study included type 2 diabetes mellitus.

The distribution of the dominant unbalanced TCM constitution types may be closely related to the pathogenesis of IGR and diabetes. In TCM, Qi indicates the refined nutritious substances constituting the human body, as well as life activities of Zang-Fu organs. In most conditions, Qi is the same as the blood in Western Medicine [19]. Qi-deficiency is defined as a lack of strength to empower the whole body, leading to dysfunction in a variety of parts of the body. The clinical manifestations include fatigue, lack of strength, shortness of breath, vacuous pulse, dizziness, blurred vision, spontaneous sweating, low voice, laziness to speak and pale tongue [20]. Many symptoms are similar to those of diabetes which are caused by lack of energy supply by glucose. Furthermore, Qi-deficiency in spleen and stomach is one important pathogenisis of obesity [21], which is a high-risk factor of metabolic syndrome and diabetes. Phlegm-damp is a constitution type of stasis of body fluid stasis and aggregation of phlegm and wetness, with common symptoms of feeling body heaviness, sticky mouth, sticky sweating, chest distress and excessive phlegm. Phlegm-damp constitution is related to many lifestyle diseases, such as hypertension, obesity, metabolic syndromes, diabetes, hyperlipidemia and stroke [22–25]. Epidemiological surveys also revealed that people with phlegm-damp constitution have a increased risk of obesity, hypertension, metabolic syndrome and diabetes than people with a balanced constitution [13]. In fact, phlegm-damp constitution is associated with many bad lifestyle behaviors, such as fatty food, barbecued food, sweet food intake and less physical activities, which are all common risk factors of metabolic syndrome and diabetes [26]. Therefore, phlegm-damp constitution could be used to estimate the risk of diabetes in IGR subjects, so as to reduce the incidence of diabetes and related complications. Damp-heat is a constitution type of internal accumulation of damp-heat, with symptoms of oily face, acne, bad breath, bitter taste in the mouth, thirsty and constipation. In TCM, spleen regulates transportation and transformation of nutrition through converting food and water into nutritions, and Damp-heat constitution was caused by disordered function of spleen and abnormal water metabolism. In Damp-heat constitution subjects, sodium elements were accumulated in intracellular fluid, leading to symptoms of edema [27], a common manifestation of diabetes and its complication, diabetic retinopathy. Therefore, Damp-heat constitution could also be used to estimate the risk of diabetes. In fact, our study showed that participants with Phlegm-damp or Damp-heat were more likely to develop diabetes in three years, and may act as independent predictive factors of diabetes.

This study we chose Phlegm-damp, Damp-heat and Qi-deficiency constitution to investigate the association of TCM body constitution and IGR. The results showed that IGR subjects with Phlegm-damp, Damp-heat or Qi-deficiency constitution all showed significantly higher serum levels of fasting plasma insulin (FPI), an indicator of insulin resistance. Furthermore, these three constitutions all showed lower serum level of adiponectin and higher serum level of leptin. Adiponectin and leptin are adipokines which are secreted from adipose tissue. In obesity, serum adiponectin is decreased while leptin is increased. Furthermore, adiponectin reduces insulin resistance while leptin enhances insulin resistance [28]. In addition, adiponectin and leptin serum concentrations may reflect adipose tissue dysfunction in IGR and might promote early pathogenetic development toward diabetes. For example, adiponectin levels were associated with macroangiopathy in IGR patients [29]. This indicates that subjects with Phlegm-damp, Damp-heat or Qi-deficiency constitution have high insulin resistance, and subsequently high risk for progression to diabetes. Our results are in consistant with other report, as evidenced by significantly lower level of serum adiponectin in patients with Phlegm-damp constitution [30]. Our results showed that IGR subjects with Phlegm-damp or Damp-heat had higher serum levels of IL-6 and TNF-α, two important inflammatory mediators. Our results are in consistant with other report that serum TNF-α, IL-6 and MCP-1 levels were significantly higher in phlegm-damp constitution population [31]. IL-6 and TNF-α are pro-inflammatory cytokines and were overproduced during obesity, thereby contributing to the pathogenesis of insulin resistance [32]. This indicates that chronic inflammation exists in population of phlegm-damp constitution. The roles of inflammation in other constitutions remain further investigation. An intersting finding of our study is that subjects with Qi-deficiency constitution showed lower serum levels of GLP-1 and GIP, two gut hormones. GLP-1 is mainly synthesized and released by L cells of the terminal ileum and colon, and GIP is mainly synthesized and released by K cells of proximal small intestine. Both GLP-1 and GIP can stimulate the secretion of insulin by pancreatic beta cells, thus increasing the plasma insulin concentration after feeding. The synthesis and secretion of GLP-1 and GIP were decreased in the presense of Insulin resistance [33]. GLP-1 and GIP can play a compensatory function of islet cell when islet cell function was gradually lost in diabetes. In fact, both two hormones are used in the treatment of type 2 diabetes, and GLP-1 can suppress insulin resistance through anti-inflammation of macrophages [34]. This indicates in IGR subjects with these three TCM constitutions, GLP-1 and GIP could be potential therapeutic tool by targeting insulin resistance and inflammatory response.

This study has several major limitations. Firstly, this is an observational study and the recruitment of IGR subjects was via rigorous random sampling method, which may have reduce the representative of our samples compared with general IGR subjects. Secondly, many other potential influencing factors, such as dietary habit, physical activities and treatments, which could also affect TCM constitutions, were not considered in the study. This may also confound the results. Thirdly, our study only suggests an association between TCM constitutions of IGR and pathogenesis and incidence of diabetes, and causal relationship cannot be made. Fourthly, our sample size is not big enough, and the role of other TCM constitutions in IGR can be investigated by enlarged sample.

## Conclusion

TCM body constitutions are important risk factors for progression to diabetes in IGR subjects, and early detection of IGR subjects who exhibit an increased risk of diabetes is crucial for preventing diabetes and its associated complications. The results of the current study show that IGR subjects with Phlegm-damp, Damp-heat or Qi-deficiency constitutions have high levels of insulin resistance and inflammatory response. IGR subjects with Phlegm-damp or Damp-heat are at a higher risk of developing diabetes, and could potentially serve as a preditor of diabetes in IGR subjects and identify these subjects for more precisive treatments. Evaluation of body constitutions by BCQ is a noninvasive and inexpensive method in clinical practice to select IGR patients who are at a high risk of diabetes..

## Appendix

The Constitution in Chinese Medicine Questionnaire.

1 = Not at all.

2 = few.

3 = sometimes.

4 = often.

5 = always.

1. Are you full of energy? 1,2,3,4,5.

2. Do you easily tired? 1,2,3,4,5.

3. Are you susceptible to shortness of breath? 1,2,3,4,5.

4. Are you susceptible to (fast heartbeat)? 1,2,3,4,5.

5. Are you susceptible to feel dizzy? Or when you stand up, you feel dizzy? 1,2,3,4,5.

6. Would you like to be quiet and lazy to talk? 1,2,3,4,5.

7. Do you have a low voice? 1,2,3,4,5.

8. Are you easy to forget things? 1,2,3,4,5.

9. Do you feel bored and depressed? 1,2,3,4,5.

10. Are you nervous and anxious? 1,2,3,4,5.

11. Do you always feel melancholy? 1,2,3,4,5.

12. Are you susceptible to feel scared or frightened? 1,2,3,4,5.

13. Do you feel chest pain? 1,2,3,4,5.

14. Do you feel chest tightness (especially in rainy and humid weather)? 1,2,3,4,5.

15. Are you susceptible to sigh without special reason? 1,2,3,4,5.

16. Do you feel your body too heavy to move? 1,2,3,4,5.

17. Do you feel your hands and feet are hot? 1,2,3,4,5.

18. Do you feel your hands and feet are cold? 1,2,3,4,5.

19. Do you feel a cold waist? 1,2,3,4,5.

20. Do you feel cold, and wear more than others? 1,2,3,4,5.

21. Do you feel the hot of your body and face? 1,2,3,4,5.

22. Do you feel that you can’t tolerate the cold in the winter than others? 1,2,3,4,5.

23. Do you feel that you are more susceptible to catch a cold than others? 1,2,3,4,5.

24. Do you sneeze even though you do not have a cold? 1,2,3,4,5.

25. Do you often have a runny nose, even if it is not a cold? 1,2,3,4,5.

26. Do you often have a stuffy nose, even if you are not a cold 1,2,3,4,5.

27. Do you feel that though slightly active or inactive, you are easy to sweat (spontaneous)? 1,2,3,4,5.

28. Do you have a sticky sweat? 1,2,3,4,5.

29. Do you find you have feet wet? 1,2,3,4,5.

30. Are you easy to be allergies (drugs, food, smell, pollen)? 1,2,3,4,5.

31. Is your skin easy to onset hives (urticaria and urticaria)? 1,2,3,4,5.

32. Is your skin allergy to appeared purpura (purple petechia) 1,2,3,4,5?

33. Is your skin often appear black imperceptibly bleeding spots (subcutaneous hemorrhage)? 1,2,3,4,5.

34. Is your skin susceptible to turn red and scratches after scratch? 1,2,3,4,5.

35. Is your skin dryness? 1,2,3,4,5.

36. Is your skin rough and delicate? 1,2,3,4,5.

37. Do you feel pain here and there? 1,2,3,4,5.

38. Is your face usually flushing or partial red? 1,2,3,4,5.

39. Is your face or nose oily or greasy? 1,2,3,4,5.

40. Is your complexion dullness? 1,2,3,4,5.

41. Are you prone to acne? 1,2,3,4,5.

42. Do you have a swollen eyes (the lower eyelids)? 1,2,3,4,5.

43. have a dark circles around the eyes.? 1,2,3,4,5.

44. Do you feel dryness of eyes? 1,2,3,4,5.

45. Do you have eye congestion (redness)? 1,2,3,4,5.

46. Do you feel dry mouth and throat? 1,2,3,4,5.

47. Do you have a feeling of blockage in the throat? 1,2,3,4,5.

48. Do you feel a bitter taste in the mouth? 1,2,3,4,5.

49. Do you have a sticky feeling in your mouth? 1,2,3,4,5.

50. Do you sleep easily? 1,2,3,4,5.

51. Do you have phlegm? 1,2,3,4,5.

52. Do you feel uncomfortable after eating or drinking cool things? Or you donnot like to have cold things? 1,2,3,4,5.

53. Do you sleep well 1,2,3,4,5.

54. Do you easily sleep? 1,2,3,4,5.

55. Are you susceptible to have loose stool? 1,2,3,4,5.

56. Do you have a sticky stool? 1,2,3,4,5.

57. Do you have a dry stool or constipation, 1,2,3,4,5.

58. Do you have a lot of urine, or a frequent micturition? 1,2,3,4,5.

59. Do you have a sense of fever in the urethra? Is your urine’s color darkness? 1,2,3,4,5.

60. Do you have decadent leucorrhea? 1,2,3,4,5.
